The article "The quality of life in patients with Parkinson's disease: Focus on gender difference" was published in 2022. Journal: Brain Behav.

# The quality of life in patients with Parkinson's disease: Focus on gender difference

**DOI:** 10.1002/brb3.2517

**Published:** 2022-02-09

**Authors:** Detao Meng, Zhaohui Jin, Lei Gao, Yixuan Wang, Ruidan Wang, Jinping Fang, Lin Qi, Yuan Su, Aixian Liu, Boyan Fang

**Affiliations:** ^1^ Parkinson Medical Center Beijing Rehabilitation Hospital Capital Medical University Beijing China

**Keywords:** gender, health‐related quality of life, Parkinson's disease, PDQ‐39

## Abstract

**Background:**

To improve understanding of gender differences on quality of life (QoL) in patients with Parkinson's disease (PWP) of a different race, the differences of clinical features and health‐related quality of life (HRQoL) between male and female PWP were studied in a small cohort early to middle stage of Chinese PWP.

**Methods:**

A cross‐sectional study was carried out. PWP were consecutively included from April 2020 to July 2021 in Beijing Rehabilitation Hospital. HRQoL, motor symptoms, and nonmotor symptoms in each patient were evaluated. The differences of demographic, motor symptoms assessments, nonmotor symptoms assessments, and QoL between two gender groups were tested using *t*‐test statistics, Mann–Whitney–Wilcoxon test, or *χ* ^2^ depending on the data type. To eliminate the possible factors contributing to the QoL, linear regression models were constructed to sort out the effect of gender.

**Results:**

One hundred and sixty‐two Parkinson's disease (PD) patients were included. Demographic, clinical characteristics, and symptom scale assessments had no statistical differences except for levodopa equivalent daily dose, Hamilton Anxiety Rating Score, REM sleep behavior disorder sleep questionnaire, and Hyposmia Rating Scale score. After baseline imbalance corrections, a significantly higher score of PD Questionnaire‐39 (PDQ‐39) in female than in male patients(*p*<.05) was found. In the questionnaire, summary Index and bodily discomfort, stigma, and emotional well‐being subscores were the main contribution differences.

**Conclusions:**

Gender differences are associated with the QoL in the early to middle stage PWP in China. Female patients have poorer QoL than male patients, especially bodily discomfort, stigma, and emotional well‐being.

## 1 INTRODUCTION

Parkinson's disease (PD) is a chronic degenerative disease characterized by motor symptoms such as bradykinesia, rest tremor, rigidity, and a variety of nonmotor symptoms, including depression, memory loss, hyposmia, and gastrointestinal and sleep dysfunction, which lead to impairment in activities of daily living and a decline in quality of life (QoL) (Meoni et al., 2020).

The epidemiology and disease manifestations of PD may differ when comparing females with males (Pavon et al., 2010). Compared with females, males have higher prevalence and incidence, earlier disease onset, more severe motor symptoms, and progression, and more frequent cognitive decline (Meoni et al., 2020). But concerning the health‐related quality of life (HRQoL), the association between sex and QoL remains controversial. A comprehensive list of gender differences in QoL in patients with Parkinson's disease (PWP) in several previous studies is displayed in Table 1 (Abraham et al., 2019; Augustine et al., 2015; Balash et al., 2019; Behari et al., 2005; Carod‐Artal et al., 2007; Dahodwala et al., 2016; Hristova et al., 2009; Kim et al., 2019; Kuopio et al., 2000; Lubomski et al., 2014; Moore et al., 2005; Yoon et al., 2017). As shown in Table 1, most of the studies show significantly better QoL of female patients than male patients (Augustine et al., 2015; Balash et al., 2019; Behari et al., 2005; Dahodwala et al., 2016; Hristova et al., 2009; Kuopio et al., 2000; Yoon et al., 2017). But some studies show no significant difference (Abraham et al., 2019; Carod‐Artal et al., 2007; Kim et al., 2019; Lubomski et al., 2014), and one study shows significantly better QoL of PD women than PD men. Furthermore, most of the research focused on Europeans, Americans, Australians, and Asians in Korea and India. To our knowledge, there are limited studies on sex differences in QoL in the Chinese PD population. The number of PWP in China accounted for approximately 23% of the entire global PD population and has a rapid increase (Collaborators GPsD, 2019). The accurate identification of gender difference is important to tailor treatment, predict prognosis, and contentment other personal and social needs in PD patients (Georgiev et al., 2017).

The article "The quality of life in patients with Parkinson's disease: Focus on gender difference" was published in 2022. Journal: Brain Behav.

**TABLE 1:** Gender differences in quality of life in Parkinson's disease in the literature

Characteristic of the study sample							
Study	Region	Sample size (M:F)	Age, mean (SD) (M:F)	Disease duration (years)	H&Y/UPDRSIII	HRQOL instrument	Gender differences
(Abraham et al., 2019)	The United States	1463 (914:549)	64.5 ± 10.4 vs 65.7 ± 11.0	n.a.	2.3 ± 0.8 vs. 2.4 ± 1.0/26.4 ± 12.4 vs. 26.3 ± 13.8	SF‐12	SF‐12 MH and SF‐12 PH: NS; females: less social support, more psychological distress, worse self‐reported disability (*p* < .05)
(Kim et al., 2019)	Korea	100 (48:52)	57.3 ± 8.5 vs 60.2 ± 6.7	10.8 ± 4.0 vs. 12.0 ± 4.7	n.a./19.6 ± 11.9 vs. 19.4 ± 11.3	SF‐36	SF‐36 score: NS; Physical‐component summary and Mental‐component summary: NS
(Balash et al., 2019)	Israel	122	68.3 ± 10.1 vs. 67.6 ± 7.7	Median: 8, IQR: 3–12 vs. median: 7.5, IQR: 3–12	Median: III, IQR: II–III/n.a.	PDQ‐39	The PDQ‐39 SI scores were higher in female patients than in male patients. Mobility as well as emotional items and pain had a greater effect on women. Cognition and communication contribute to worsened QoL more in men than in women
(Yoon et al., 2017)	Korea	89 (47:42)	68.18 ± 8.14 vs. 68.90 ± 7.71	2.6 ± 2.8 vs. 3.2 ± 3.6	2.1 ± 0.9 vs. 2.1 ± 0.9/24.2 ± 13.2 vs. 22.9 ± 12.9	PDQ‐39	The PDQ‐39 SI scores were higher in female patients than in male patients (*p* < .05)
(Dahodwala et al., 2016)	Canada, the Netherlands, Israel, the United States	4679 (2938:1741)	65.5 ± 9.7 vs. 66.9 ± 9.7	8.7 ± 6.0 vs. 8.9 ± 6.6	Range: 1–5/n.a.	PDQ‐39	The PDQ‐39 SI scores were higher in female patients than in male patients. Men reported lower QoL in mobility, emotional, and pain
Augustine et al., 2015	The United States and Canada	1738 (617:1121)	n.a.	3.2 ± 2.0 vs. 3.3 ± 2.3	n.a./18.2 ± 8.2 vs. 17.0 ± 8.6	PDQ‐39	The PDQ‐39 SI scores were higher in female patients than in male patients
(Lubomski et al., 2014)	Australia	210 (129:81)	70.1 ± 10.4 vs. 67.6 ± 11.3	7.4 ± 5.7 vs. 7.0 ± 5.8	n.a./27 ± 13 vs. 23 ± 13	PDQ‐39	The PDQ‐39 SI scores: NS. The PDQ‐39 showed men reported lower QoL in activities of daily living, cognition, and communication subscales (*p* < .05)
(Hristova et al., 2009)	Bulgaria	866 (412:454)	74.0 ± 0.3 vs. 73.5 ± 0.4	6.7 ± 0.9	Range: 1−5/n.a.	PDQ‐39	Significantly poorer QoL of women than men. Female PD patients: significantly worse assessment of QoL in aspects mobility, emotional well‐being, social support, and bodily discomfort
(Carod‐Artal et al., 2007)	Brazilian	144 (77:67)	60 ± 11.4 vs. 64 ± 10.6	6.6 ± 3.8	Median: 2, IQR: 1.5−2.5/27.9 ± 14.5	PDQ‐39	The PDQ‐39 SI scores: NS; female: worse mobility, emotional well‐being, cognition, and bodily discomfort
(Moore et al., 2005)	Israel	124 (69:55)	65.8 ± 10.2	8.5 ± 5.8	2.7 ± 0.9/48.4 ± 17.2	PDQ‐39	Significantly better QoL of PD women than PD men
(Behari et al., 2005)	India	278 (218:60)	58.3 ± 10.5 vs. 53.1 ± 10.8	4.7 ± 3.8 vs. 4.4 ± 4.4	n.a./n.a.	PDQL	Women scored significantly lower on parkinsonian symptoms, systemic symptoms, social symptoms, emotional symptoms, and total score
(Kuopio et al., 2000)	Finland	228 (104:124)	71.3 ± 9.5 vs. 73.4 ± 8.4	8.2 ± 5.1 vs. 9.5 ± 5.7	2.6 ± 0.9/n.a.	SF‐36	Women scored significantly lower on five dimensions (physical functioning, role limitations—physical, social functioning, bodily pain, and mental health)

Abbreviations: n.a., not available; NS, not significant; M:F, MALE:FEMALE; PDQ‐39 SI, PDQ‐39‐Summary Index; PDQ‐39, PD Questionnaire‐39; PDQL, Parkinson disease quality of life questionnaire; SF‐12, 12‐Item Short Form Health Survey; SF‐36, 36‐Item Short Form Health Survey.

The article "The quality of life in patients with Parkinson's disease: Focus on gender difference" was published in 2022. Journal: Brain Behav.

Therefore, we sought to evaluate the gender differences in QoL in a Chinese PD population. Meanwhile, we also evaluated the differences in clinical features, such as motor and nonmotor symptoms.

## 2 METHODS

### 2.1 Study population

A cross‐sectional study was performed on consecutive PWP attending our inpatient rehabilitation in Beijing Rehabilitation Hospital from April 2020 to July 2021. Inclusion criteria were as follows: (1) idiopathic PD diagnosed by a neurologist according to the Movement Disorder Society criteria (Postuma et al., 2015), (2) Hoehn and Yahr (H&Y) stage: I–III stages, (3) no deep brain stimulation or in vivo implantation treatment, and (4) were able to understand each item of the informed consent and willing to sign the informed consent. Exclusion criteria were as follows: (1) secondary or atypical parkinsonism such as multiple system atrophy, corticobasal degeneration, and progressive supranuclear palsy, (2) serious medical conditions, for example, severe infection, malignancy, anemia, or hepatic disease, (3) individuals with dementia or severe psychiatric symptoms. This study was approved by the ethics committee of the Beijing Rehabilitation Hospital. All participants signed informed consent following the Declaration of Helsinki. Clinical and demographic data collected included age, age at diagnosis, gender, education years, body mass index, and disease duration. In addition, the levodopa equivalent daily dose (LEDD) was calculated.

### 2.2 Clinical assessments

The Movement Disorder Society‐Sponsored Revision of the Unified Parkinson's Disease Rating Scale (MDS‐UPDRS) was used to assess PD motor functions (C. G. Goetz et al., 2007), and the H&Y stage was used to assess clinical stage (Hoehn & Yahr, 1967). The MDS‐UPDRS consists of part I—nonmotor experiences of daily living, part II—motor experiences of daily living, part III–a disease‐relevant motor examination, and part IV–motor complications (C. Goetz et al., 2008). MDS‐UPRDS part III was further divided into four subscores: tremor (items 3.15−18), rigidity (3.3), bradykinesia (3.4−8, 3.14), and axial signs (3.1–2, 3.9−13). MDS‐UPRDS part IV was further divided into two subscores: dyskinesia (4.1−4.2) and motor fluctuations (4.3−4.6) (Kuhlman et al., 2019).

Nonmotor symptoms were evaluated using the following scales: Montreal Cognitive Assessment (MoCA) for cognitive function, Hamilton Depression Rating Scale (HAMD) for depression (Hamilton, 1960); Hamilton Anxiety Rating Scale (HAMA) for anxiety (Hamilton, 1959); REM sleep behavior disorder sleep questionnaire (RBDSQ) for REM sleep behavior disorder (Li et al., 2017); Parkinson Fatigue Scale (PFS⁃16) for fatigue (Brown et al., 2005); Parkinson's Disease Sleep Scale score (PDSS) for the severity of sleep disturbances (Chaudhuri et al., 2002); Hyposmia Rating Scale (HRS) for assessing olfactory function (Millar Vernetti et al., 2012); Modified Apathy Evaluation Scale (MAES) for apathy (Starkstein et al., 1992); and questionnaire for impulsive‐compulsive disorders in Parkinson's disease (QUIP) for impulsive‐compulsive disorders (Weintraub et al., 2009), Patient Assessment of Constipation Quality of Life (PAC‐QOL) questionnaire for constipation (Marquis et al., 2005).

The article "The quality of life in patients with Parkinson's disease: Focus on gender difference" was published in 2022. Journal: Brain Behav.

The PD Questionnaire‐39 (PDQ‐39) was used to evaluate patients’ HRQoL. PDQ‐39 is a validated disease‐specific HRQoL measure in PD (Neff et al., 2018). It includes eight dimensions assessing problems with mobility, activities of daily living, emotional well‐being, stigma, social support, cognition, communication, and bodily discomfort. Each item of the PDQ‐39 is scored on a five‐point scale from “never” to “always.” PDQ‐39 subscale scores and the PDQ‐39 summary index (SI) range from 0 to 100 (Jenkinson et al., 1997). A higher score means a poorer QoL.

### 2.3 Statistical analysis

All data except for the marital status are expressed as mean ± SD. Marital status was reported in terms of percentage. Data distribution and normality were evaluated with the Shapiro–Wilk test. The Mann–Whitney–Wilcoxon test was used to compare age at diagnosis, education years, disease duration, LEDD, H&Y stage, UPDRS part I score, UPDRS part IV score, tremor subscore, rigidity subscore, bradykinesia subscore, axial subscore, dyskinesia score, motor fluctuations score, MoCA, HAMA, HAMD, RBDSQ, PFS⁃16, PDSS, HRS, MAES, QUIP, PAC‐QOL, PDQ‐39‐SI, bodily discomfort, communication, cognition, social support, stigma, emotional well‐being, activities of daily living, and mobility. Independent‐samples *t*‐tests were used to analyze age, body mass index, and UPDRS parts II and III scores. Differences in proportions of marital status as categorical variables were analyzed using *χ* ^2^ test. Linear regression models were constructed to evaluate the effect of gender differences on PDQ‐39‐SI after controlling for HAMA, LEDD, RBDSQ, and HRS. We considered *p* < .05 to be statistically significant. These statistical data were analyzed using SPSS version 21 (SPSS Inc., Chicago, IL, USA).

## 3 RESULTS

A total of 162 (70 males and 92 females) PWP were included. The demographics for 162 PWP are shown in Table 2. We did not observe differences between male and female patients in age, age at PD diagnosis, education years, body mass index, disease duration, and marital status. Male patients had higher LEDD compared to female patients (*p*<.05).

The article "The quality of life in patients with Parkinson's disease: Focus on gender difference" was published in 2022. Journal: Brain Behav.

**TABLE 2:** Demographic of the Parkinson's disease

Variables	PD (M = 70)	PD (F = 92)	*p*‐Value
Age	60.41 (9.23)	59.60 (7.24)	.529^a^
Age at diagnosis	53.91 (9.58)	52.21 (7.99)	.618^b^
Education years	12.87 (3.71)	12.14 (3.64)	.189^b^
BMI (kg/m^2^)	24.06 (2.71)	23.49 (3.00)	.327^a^
Disease duration, years	6.56 (3.91)	6.38 (3.92)	.698^b^
LEDD (mg/d)	592.58 (280.23)	501.18 (216.96)	.022^b*^
Marital status, *n* (%)			.47^c^
Married	66 (94.29%)	86 (93.48%)	
Single	1 (1.43%)	0 (0%)	
Divorced/separated	1 (1.43%)	2 (2.17%)	
Widowed	2 (2.86%)	4 (4.35%)	

*Note*: Data are presented as the mean (SD) except for the marital status. Marital status was reported as *n* (%). a: independent‐samples *t*‐tests; b: the Mann–Whitney–Wilcoxon test; c: *χ* ^2^ test.

Abbreviations: BMI, body mass index; LEDD, levodopa equivalent daily dose; PD, Parkinson's disease.

*p < .05.

The clinical characteristics and symptom scale assessments for 162 PWP are shown in Table 3. We did not observe differences between male and female PWP in the H&Y stage, UPDRS parts I, II, III, and IV scores, tremor subscore, rigidity subscore, bradykinesia subscore, axial subscore, dyskinesia score, motor fluctuations score, MoCA, HAMD, PFS‐16, PDSS, MAES, QUIP, and PAC‐QOL. Male patients had a higher RBDSQ score (*p*<.05) and lower HAMA and HRS scores (*p*<.05) compared to female patients.

**TABLE 3:** Clinical characteristics and symptom scale assessments

Assessment	PD (M = 70)	PD (F = 92)	*p*‐Value
Motor symptoms			
Hoehn & Yahr stage, *n* (%)			.678^b^
1	1 (1.43%)	2 (2.17%)	
1.5	6 (8.57%)	8 (8.70%)	
2	27 (38.57%)	44 (47.83%)	
2.5	21 (30.00%)	19 (20.65%)	
3	15 (21.43%)	19 (20.65%)	
UPDRS part II score	11.53 (6.25)	10.88 (6.74)	.539^a^
UPDRS part III score	33.86 (13.32)	32.70 (13.08)	.658^a^
UPRDS part IV score	3.34 (3.52)	3.90 (3.62)	.314^b^
Tremor subscore	4.70 (4.86)	4.22 (4.06)	.675^b^
Rigidity subscore	9.51 (3.07)	9.02 (3.08)	.276^a^
Bradykinesia subscore	14.37 (7.22)	14.61 (6.95)	.822^a^
Axial subscore	6.88 (3.26)	6.71 (3.79)	.558^b^
Dyskinesia score	0.27 (0.66)	0.37 (0.90)	.834^b^
Motor fluctuations score	2.45 (2.64)	3.20 (3.01)	.216^b^
Nonmotor symptoms			
UPDRS part I score	9.66 (6.43)	9.57 (5.05)	.597^b^
MoCA	25.18 (3.43)	25.13 (5.11)	.468^b^
HAMA	9.651 (6.75)	12.04 (6.71)	.043^b*^
HAMD	7.18 (5.00)	9.33 (6.31)	.117^b^
RBDSQ	4.34 (3.85)	2.52 (2.36)	.010^b*^
PFS‐16	44.51 (15.30)	44.06 (13.89)	.739^a^
PDSS	108.28 (28.87)	107.92 (27.15)	.765^b^
HRS	15.62 (6.48)	17.93 (5.76)	.026^b*^
MAES	12.02 (7.83)	12.73 (7.99)	.654^b^
QUIP	11.38 (18.17)	7.31 (13.54)	.449^b^
PAC‐QOL	55.29 (19.55)	50.53 (18.66)	.134^b^

*Note*: Data are presented as the mean (SD) except the marital status. Marital status was reported as *n* (%). a: independent‐samples *t*‐test; b: the Mann–Whitney–Wilcoxon test, c *χ* ^2^ test.

The article "The quality of life in patients with Parkinson's disease: Focus on gender difference" was published in 2022. Journal: Brain Behav.

Abbreviations: HAMA, Hamilton Anxiety Rating Scale; HAMD, Hamilton Depression Rating Scale; HRS, Hyposmia Rating Scale; MAES, Modified Apathy Evaluation Scale; MoCA, Montreal Cognitive Assessment; PAC‐QOL, Patient Assessment of Constipation Quality of Life questionnaire; PD, Parkinson's disease; PDSS, Parkinson's Disease Sleep Scale score; PFS ⁃ 16, Parkinson Fatigue Scale; QUIP, questionnaire for impulsive‐compulsive disorders in Parkinson's disease; RBDSQ, REM sleep behavior disorder sleep questionnaire; UPDRS, Unified Parkinson's Disease Rating Scale.

*p < .05.

Gender differences impact on PD patient's QoL according to PDQ‐39 is shown in Table 4. We did not observe differences between male and female PWP in communication, cognition, social support, activities of daily living, and mobility. Differences in HRQoL were observed, with female patients demonstrating higher scores compared to male patients on PDQ‐39‐SI (*p* < .05). Furthermore, female patients had a higher score compared to male patients on bodily discomfort, stigma, and emotional well‐being (*p* < .05). Gender differences impact on PD patient's PDQ‐39 domains is shown in Figure 1.

**TABLE 4:** Gender differences impact on Parkinson's disease (PD) patient's quality of life according to PD Questionnaire‐39 (PDQ‐39)

PDQ‐39 domains	PD (M = 70)	PD (F = 92)	*p*‐Value
PDQ‐39‐SI	20.07 (10.70)	25.86 (12.49)	.010^*^
Bodily discomfort	22.50 (21.95)	34.78 (20.25)	.000^*^
Communication	13.45 (18.02)	12.05 (15.89)	.889
Cognition	25.09 (18.29)	28.06 (15.15)	.271
Social support	6.90 (16.96)	9.69 (19.50)	.314
Stigma	22.77 (19.91)	31.52 (25.29)	.035^*^
Emotional well‐being	21.13 (17.13)	27.81 (17.15)	.008^*^
Activities of daily living	16.84 (13.69)	15.12 (14.61)	.286
Mobility	21.36 (13.99)	27.26 (19.35)	.103

*Note*: Data are presented as the mean (standard deviation). All data were analyzed by the Mann–Whitney–Wilcoxon test.

^*^ *p* < .05.

**FIGURE 1:** Polar plot for the different PDQ‐39 domains depending on gender differences. Female patients had higher scores compared to male patients on bodily discomfort, stigma, and emotional well‐being (*p*<.05). Abbreviations: ADL, activities of daily living; PDQ‐39, Parkinson's disease Questionnaire‐39

Multiple linear regression models of HRQoL scales are shown in Table 5. Sex, LEDD, RBDSQ, HRS, and HAMA were included as independent variables. Sex still had a strong influence on HRQoL after controlling for HAMA, LEDD, RBDSQ, and HRS.

**TABLE 5:** Multiple linear regression models of health‐related quality of life (HRQoL) scales

Variables	Standardized *β*	*t*	Significance
Sex	.26	2.37	.020^*^
LEDD	.02	0.17	.866
RBDSQ	.18	1.71	.090
HRS	.02	0.20	.842
HAMA	.31	3.14	.002^*^

Abbreviations: HRS, Hyposmia Rating Scale; HAMA, Hamilton Anxiety Rating Scale; LEDD, levodopa equivalent daily dose; RBDSQ, REM sleep behavior disorder sleep questionnaire.

^*^ *p* < .05.

The article "The quality of life in patients with Parkinson's disease: Focus on gender difference" was published in 2022. Journal: Brain Behav.

## 4 DISCUSSION

The present study demonstrates that gender differences are associated with the QoL in the Chinese PD population. Female patients have poorer QoL than male patients, especially bodily discomfort, stigma, and emotional well‐being. This research filled some important gaps in our knowledge regarding sex differences in QoL in the Chinese PD population. Furthermore, we found that males had a higher RBDSQ score and lower HAMA and HRS scores compared to females.

It is thought that PD had a comprehensive impact on HRQoL and was impaired very early. Carod‐Artal et al. (2007) found that PD can affect all HRQoL measures since the first stages of the disease and HRQoL gradually deteriorate with the disease progresses in Brazilian patients, but they did not find gender differences impact on QoL. Meanwhile, another three studies reach the same conclusions (Abraham et al., 2019; Kim et al., 2019; Lubomski et al., 2014). Lubomski et al. suggested that although the PDQ‐39 SI scores have no significant differences, men reported lower QoL in activities of daily living, cognition, and communication sub‐scales (*p* < .05) in Australia. Abraham et al. (2019) use the patient‐reported 12‐Item Short‐Form Health Survey (SF‐12) to assess HRQoL in a US population. They found that compared to male patients, female patients reported poorer HRQoL scores, and female patients had significantly less social support, more psychological distress, and worse self‐reported disability. Kim et al.’s study mainly assessed the influence of sex on the effects of subthalamic nucleus stimulation. At baseline, SF‐36 score, physical‐component summary and mental‐component summary all have no significant difference in South Koreans. In addition, Moore et al. suggested significantly better QoL of PD women than PD men in Israel.

On the other hand, more research suggested male patients’ QoL better than female patients. Yoon et al. (2017) found female patients have poorer QoL than male patients in other South Koreans. Balash et al. suggested that the PDQ‐39 SI scores were higher in female patients than male patients. Mobility, emotional, and pain items had a greater effect in women, and cognition and communication contribute to worsened QoL more in men than in women in another Israel population (Balash et al., 2019). Dahodwala et al. also found male patients’ QoL better than female patients. Female patients reported lower QoL in mobility, emotional, and pain in a National Parkinson's Outcomes Project including Canada, Netherlands, Israel, and the United States (Dahodwala et al., 2016). Augustine et al. (2015) found that the PDQ‐39 SI scores were higher in female patients than in male patients in early treated PD of North America. Hristova et al. (2009) and Kuopio et al. (2000) both found significantly poorer QoL of women than men in Europe. Hristova et al. (2009) report that female PD patients have a significantly worse assessment of QoL in mobility, emotional well‐being, social support, and bodily discomfort in Bulgaria. Kuopio et al. (2000) report that women scored significantly lower on five dimensions (physical functioning, role limitations—physical, social functioning, bodily pain, and mental health) in Finland. Meanwhile, Behari et al. (2005) found female patients’ QoL better than male patients in India. Females reported lower QoL in parkinsonian symptoms, systemic symptoms, social symptoms, and emotional symptoms.

The article "The quality of life in patients with Parkinson's disease: Focus on gender difference" was published in 2022. Journal: Brain Behav.

Through literature review, we found that the association between sex and QoL remains controversial, and different patient groups may have different manifestations of QoL. According to the Prevalence of Parkinson's Disease report, the number of PWP is 3.62 million in China (Qi et al., 2021) and 50% of global PD patients will be Chinese by 2030 (Dorsey et al., 2007), but few studies focus on the QoL in PWP in the Chinese population. Hu et al. (2018) and Song et al. (2014) explored the determinants of QoL in a Southwest Chinese PD population. They both found that gender is a determinant of QoL in the Chinese PD population. Tao Hu et al.’s study focused on exploring the gender and onset age‐related nonmotor symptoms profiles and the determinants of QoL in drug‐naïve PD patients (Hu et al., 2018). Song et al.’s study focused on the association between nonmotor symptoms and HRQoL in the Chinese PD population (Song et al., 2014). To our knowledge, this is the first study that mainly focuses on the effects of gender differences on QoL in a Chinese PD population and all the patients in the early to middle stage. Consisting with previous studies (Augustine et al., 2015; Balash et al., 2019; Behari et al., 2005; Dahodwala et al., 2016; Hristova et al., 2009; Kuopio et al., 2000; Yoon et al., 2017), We found that female patients have poorer QoL than male patients. Further subclass analysis of the PDQ‐39 suggested that female patients have higher scores in bodily discomfort, stigma, and emotional well‐being. Gender differences on QoL in Chinese PD population are similar to other regions’ study. Our study has important implications for improving care and outcomes for female patients in China. We should use different patient management strategies between male and female PD patients.

The article "The quality of life in patients with Parkinson's disease: Focus on gender difference" was published in 2022. Journal: Brain Behav.

Apart from QoL, we also found that male patients had a higher RBDSQ score and lower HAMA and HRS scores compared to female patients. So far, the incidence of RBD is also controversial in different studies. some studies reported a higher prevalence in male PD patients than in female patients (Ozekmekci et al., 2005; Yoritaka et al., 2009), but some studies reported opposite results (Bjornara et al., 2013; Bugalho et al., 2011). We found that male patients had higher RBDSQ scores compared to female patients. At the same time, our study showed that male patients had lower HRS scores compared to female patients, suggesting that men have worse olfactory function than women consistent with the previous study (Picillo et al., 2013). Meanwhile, we also found that females experienced higher anxiety than male patients consistent with the previous study (Leentjens et al., 2011; Liu et al., 2015).

Why do male patients have better QoL than female patients? Anxiety may be one possible reason. Anxiety frequently afflicts PWP and negatively impacts their QoL, especially female patients (D'Iorio et al., 2017; Dissanayaka et al., 2014; Pontone et al., 2019). As we described above, anxiety was more severe in female patients than in male patients in our research. Moreover, Kuhlman et al.’s research considered that anxiety, depression, excessive daytime sleepiness, and apathy were independently associated with worse HRQoL (Kuhlman et al., 2019). Santos et al.’s research considered mood, and nonmotor symptoms burden seems to be the most relevant factors affecting patients’ QoL with PD (Santos Garcia et al., 2019). Although our male patients had more severe RBD symptoms, female patients experienced more severe anxiety, depression, and apathy symptoms than male patients, and anxiety and depression were recognized as more important than other factors in determining the QoL of PWP (Rahman et al., 2008). Finally, as shown in other studies (Behari et al., 2005; Hristova et al., 2009), female patients’ poor QoL may be a result of their more active participation in everyday household activities such as cooking, increasing concern for poor performance. There is substantial research showing that women do more housework than men in East Asian countries (Hu & Mu, 2021; Midgette, 2020; Oshio et al., 2012). Therefore, although our study did not assess the participation of female patients in housework, we still considered it as a possible reason why the QoL of female patients is lower than that of men.

Our study has several limitations. First, we included only PD patients rated between 1 and 3 on the H&Y stage, which might lead to selection bias. Because the study participants were all Chinese population, the generalizability of these observations across the different countries should be verified. Second, the economic status of patients may have a certain impact on their QoL, our study did not include it. Finally, we conducted a small sample data study and further studies are required before they can be used for clinical management or planning of patient care.

The article "The quality of life in patients with Parkinson's disease: Focus on gender difference" was published in 2022. Journal: Brain Behav.

In conclusion, the present study shows that gender differences are associated with the QoL in PD patients. Female patients have poorer QoL than male patients, especially bodily discomfort, stigma, and emotional well‐being. When we manage female PD patients, we should pay more attention to bodily discomfort, stigma, and emotional well‐being for improving the QoL and inform the family members and caregivers to actively participate in the daily family activities to reduce the living burden of patients, and reduce the psychological burden of patients through positive psychological counseling and health education.

## CONFLICT OF INTEREST

The authors declare no conflict of interest.

### PEER REVIEW

The peer review history for this article is available at https://publons.com/publon/10.1002/brb3.2517

## Data Availability

The data of this study are available from the corresponding author upon request.
